# Influence of Degree of Chinese Cultural Identity and Performance Expectation on Consumption Attitude for Health Care of Traditional Chinese Medicine

**DOI:** 10.1155/2022/3342169

**Published:** 2022-06-01

**Authors:** Shengliang Lin, Yan Yan, Chenxi Hu

**Affiliations:** ^1^School of Journalism and Communication, Jinan University, Guangzhou 510632, China; ^2^College of Applied Arts and Science, Beijing Union University, Beijing 100191, China

## Abstract

There are some advantages of traditional Chinese medicine in anti-COVID-19, and more and more Chinese people are beginning to accept health care of Traditional Chinese Medicine (TCM). By selecting two important independent variables, degree of Chinese cultural identity and performance expectation, their influence mechanism on the consumption attitude of health care for TCM is studied. The results show that the two dimensions of degree of Chinese cultural identity significantly affect the consumption attitude of health care for TCM, and the surface recognition dimension negatively affects the behavioral attitude of health care for TCM. The deep behavioral dimension has a positive impact on the consumption attitude of health care for TCM. Performance expectation has a positive impact on the consumption attitude of health care for TCM. Chinese cultural identity and performance expectation have a positive interaction on the consumption attitude of health care for TCM.

## 1. Introduction

The theory of TCM originates from philosophy, so TCM cannot accurately clarify the anatomical structure, physiological function and pathological changes of the human body in detail. TCM advocates experience accumulation and reasoning in research methods. This makes many people think that TCM is generally a summary of intuitive experience, and its diagnosis and treatment methods do not rely on many instruments and equipment. However, TCM emphasizes “individualized” treatment, that is, the same disease occurs in different people, and different methods of scientific treatment are selected in combination with the patient's own conditions. It is the foundation for TCM to remain invincible. Health care of Traditional Chinese Medicine (TCM) refers to a kind of medical activity to take care of life, enhance physique and prevent diseases through various methods, to prolong life. It focuses on integrity and systematicness. The purpose is to prevent diseases in advance. The items of health care TCM generally include diet therapy, pharmacotherapy, acupuncture, cupping, massage, etc.

The research on health care and health communication of traditional Chinese medicine is the combination of communication with traditional Chinese medicine theory and traditional Chinese medicine culture. It is the localized development of health communication. With China's economic development and changes in social structure, people's health awareness is increasing, and the demand and consumption of traditional Chinese medicine health care are also growing. COVID-19 has made many Chinese realize the importance of health and immunity. More and more Chinese people are beginning to accept health care of Traditional Chinese Medicine (TCM). They consider that compared with material wealth, physical health and hobbies can better define success [1]. If physical health is zero, no matter how good it is in other aspects, it is meaningless. It can be said that the improvement of health awareness has further changed people's consumption attitude towards health care of health care of TCM, and the concept of “prevention of disease” of front-end health care and prevention is deeply rooted in the hearts of the people. Compared with western developed countries, China's health industry is still in the primary stage of development. The consumption market of health care health care of TCM has great potential and unlimited space.

Health care of traditional Chinese medicine has its unique industrial advantages. Shao believes that TCM is the epitome of Chinese culture and the “golden key” to open the palace of Chinese culture [2]. Moreover, Chinese culture has also nurtured the health care industry of TCM, contributing to the organic combination of the two. Pan explored the recognition of TCM culture by audiences of different ages in the new era and found that most of the public have a relatively high level of recognition of TCM culture [3]. Huang et al. believe that in the modern consumption mode, individuals will consume goods consistent with their recognized culture, and pursue a sense of belonging by consuming goods matching the culture of collective identity [4]. Therefore, the health care industry of TCM has the dual attributes of material and culture.

Venkatesh et al. proposed the “Unified Theory of Acceptance and Use of Technology” (“UTAUT”). It includes four main dimensions: Performance expectation (refers to the expected help degree that individuals feel they have achieved by using the service); Effort impact (refers to the degree of effort required by individuals to use the service); Social impact (refers to the degree of influence by social groups that individuals can feel); Promotion factors (refers to the degree of support that individuals feel) [5]. This model is widely used in the field of consumer behavior. The research of Zhou et al. shows that social impact has the greatest impact on the sustainable use intention of consumers of light food products, followed by promotion factors, performance expectations and product factors, and effort has the weakest impact [6]. The results of Ye et al. show that performance expectation, effort expectation, brand loyalty and social impact have a significant positive impact on consumers' willingness to use cross-border products [7]. Through structural equation model. Yang showed that performance expectation has a positive impact on the willingness of the elderly to use the health management system [8]. The above research shows that performance expectation is one of the important variables affecting consumption attitude. Although there are other variables, performance expectation plays the most important role in terms of health care for TCM.

In COVID-19, TCM plays a very important role in helping patients' treatment and prevention. This shows that in the face of diseases, the integration of TCM and Western medicine has great practical significance. As one of the quintessence of Chinese civilization, TCM is the essence of disease treatment and health care. This understanding will contribute to the recovery of TCM health care market rapidly. In short, the study of consumer behavior has industry differences. When selecting relevant variables, we should select the corresponding variables to process the model construction. In today's society, staying up late, staying sedentary and fast food have become important factors affecting people's health. Although people have great demand for traditional Chinese medicine of health care, they may have different recognition of Chinese culture under the baptism of market economy. Therefore, this paper selects two important independent variables, degree of Chinese cultural identity and performance expectation, to study their impact on the consumption attitude of health care for TCM.

## 2. Theoretical Framework and Research Hypotheses

Schneider and Shiffrin put forward the “Double Processing Theory”. According to this theory, human cognitive processing can be divided into two categories: automatic processing and controlled processing. Automatic processing is not limited by cognitive resources. It does not need to be noticed. It is carried out automatically. Automatic processing processes are triggered by appropriate stimulation, occur relatively quickly, and do not affect other processing processes. Due to the limitation of cognitive resources, the processing process of controlled processing is difficult to change after acquisition or formation. The participation that needs attention can be continuously adjusted with the change of cultural environment. The effectiveness of this theory has been widely supported by research [9].

“Dual Processing Theory” further points out two separate processing: associative processing and rule-based processing. Associative processing corresponds to automatic processing. It depends on many connections, which are based on the repetition of related events. These processes are relatively autonomous operations and require less memory resources. Rule-based processing correspond to controlled processing. It relies on symbolization and uses certain rules to solve problems, which has a great demand for memory [10–12]. In this paper, Chinese cultural identity is controlled processing, which is rule-based processing; Performance expectation is automatic processing, which is based on associative processing. Based on the “Dual Processing Theory”, this paper investigates the influence mechanism of Chinese cultural identity and performance expectation on the consumption attitude of health care for TCM.

Wang believes that consumption has distinct symbolism, and there is an interactive relationship between cultural identity and symbolic consumption [13]. Wu found that Chinese identity has a significant positive effect on the consumption intention of medicated diet [14]. Therefore, this paper puts forward the following assumptions.

H_1_: The degree of Chinese cultural identity has a positive impact on the consumption attitude of health care for TCM.

H_1-1_: The degree of Chinese cultural identity has a positive impact on the cognitive attitude of health care for TCM.

H_1-2_: The degree of Chinese cultural identity has a positive impact on the emotional attitude of health care for TCM.

H_1-3_: The degree of Chinese cultural identity has a positive impact on the behavioral attitude of health care for TCM.

Guo found that performance expectations, contributing factors, effort expectations, social impact and consumer innovation have a positive impact on College Students' willingness to use internet credit products [15]. The research of Li shows that performance expectation, social impact, perceived risk and perceived trust have a significant effect on users' choice intention. The positive impact of performance expectation on users' choice intention of internet financial products is very significant [16]. Therefore, this paper puts forward the following assumptions.

H_2_: Performance expectation has a positive impact on the consumption attitude of health care for TCM.

H_2-1_: Performance expectation has a positive impact on the cognitive attitude of health care for TCM.

H_2-2_: Performance expectation has a positive impact on the emotional attitude of health care for TCM.

H_2-3_: Performance expectation has a positive impact on the behavioral attitude of health care for TCM.

Ikram found that performance expectation, hedonic motivation, habit and perceived credibility are the antecedents of behavior tendency, while the five dimensions of culture (collectivism, uncertainty avoidance, power distance and time tendency) have a significant regulatory effect on the relationship between antecedents and behavior tendency [17]. Therefore, this paper puts forward the following assumptions.

H_3_: The degree of Chinese cultural identity and performance expectation interact with the consumption attitude of health care for TCM.

H_3-1_: Degree of Chinese cultural identity and performance expectation interact with the cognitive attitude of health care for TCM.

H_3-2_: Degree of Chinese cultural identity and performance expectation interact with the emotional attitude of health care for TCM.

H_3-3_: Degree of Chinese cultural identity and performance expectation interact with the behavioral attitude of health care for TCM.

## 3. Research Design

### 3.1. Research Framework

On the basis of theoretical analysis and research assumptions, we propose the influencing factor model of TCM health care consumption attitude, as shown in Figure 1.

### 3.2. Operational Definition

This paper refers to the Chinese Cultural Identity Scale formulated by Phinney and Li, the Performance Expectation Scale formulated by Venkatesh and the Consumer Attitude Scale formulated by Mitchell and Olsen [4, 18–20]. We fine tune the former related scales in combination with the characteristics of health care in the traditional Chinese medicine to obtain the following variables: degree of Chinese cultural identity, performance expectation, cognitive attitude, emotional attitude and behavioral attitude. The operational definition of five variables of behavior and attitude is shown in Table 1.

### 3.3. Research Methods

This paper adopts the method of questionnaire survey. The sample size of the questionnaire is generally 10 times or more than the total number of items in the questionnaire. In this formal survey, 800 questionnaires were distributed through snowball sampling. 784 valid questionnaires and 16 invalid questionnaires were recovered. The effective questionnaire achievement rate was 98.00%, which met the requirements. The demographic characteristics of the sample are shown in Table 2. The sample size distribution of gender, age, educational background, average monthly consumption and occupation is relatively reasonable. This paper will use the following statistical methods for data analysis: factor analysis and structural equation model analysis. Spss28.0 is adopted to process the data.

## 4. Data Analysis and Model Validation

### 4.1. Initial Model

Through preliminary exploratory factor analysis, this paper finds that there are two dimensions of Chinese national identity: surface cognition (Q1 - Q10) and deep behavior (Q11 - Q18). According to the operational definition, theoretical model and research hypothesis, the initial model diagram of six variables including degree of Chinese cultural identity (surface cognition and deep behavior), performance expectation, cognitive attitude, emotional attitude and behavioral attitude is constructed, as shown in Figure 2.

### 4.2. Test of Reliability and Validity

This paper adopts *α* Coefficient to measure the reliability of the scale, when the *α* Coefficient is higher than 0.70, it is considered that the credibility and stability of the scale meet the requirements. Through confirmatory factor analysis (Table 3), we found that the reliability of surface cognition, deep behavior, performance expectation, cognitive attitude, emotional attitude and behavioral attitude were 0.951, 0.918, 0.972, 0.807, 0.882 and 0.850, respectively, all above 0.7. The overall *α* Coefficient for the reliability of the questionnaire was 0.964, indicating that the reliability of the questionnaire is good. The reliability coefficients of each variable and its measurement dimensions in this study are within a reasonable range. The questionnaire has high consistency and stability, and the reliability of the scale is guaranteed.

Confirmatory factor analysis can also test convergent validity and discriminant validity. The criteria for judging the convergence validity are as follows: the absolute value of the estimated value of factor load should be more than 0.5, and the best index value should be more than 0.7; The index value of average variance extraction (AVE) should be above 0.5; The construct reliability index value should be higher than 0.7. The data show that they all meet the requirements, indicating that the questionnaire has good convergent validity. The criterion to judge the discriminant validity is whether the square root of AVE is higher than the correlation coefficient between the two factor constructs. The data show that the square roots of AVE of surface cognition, deep behavior, performance expectation, cognitive attitude, emotional attitude and behavioral attitude are 0.770, 0.753, 0.764, 0.825, 0.837 and 0.776, respectively, which are greater than their corresponding correlation coefficients, indicating that the questionnaire has good differential validity.

### 4.3. Structural Equation Model and Hypothesis Test

#### 4.3.1. Fitting Test of Model

It can be seen from Table 4 that the GFI, AGFI, NFI, CFI, TLI and IFI indexes of the model meet the ideal standard, the Chi Square/DF value is 2.941 (less than 5), which is ideal. The RMSEA is 0.071 (less than 0.08). On the whole, the model fits well and the fitting results are good.

#### 4.3.2. Path Analysis

The path analysis is shown in Table 5.

#### 4.3.3. Modified Model

According to the above analysis and results, we modified the structural equation model, as shown in Figure 3. From the Figure, we can see that the hypotheses of H_2_ and H_3_ are proved, while H_1_ and its sub-hypotheses are rejected. Among them, the surface cognitive dimension of degree of Chinese cultural identity does not significantly affect the cognitive attitude and emotional attitude of health care in the traditional Chinese medicine, while the surface cognitive dimension of degree of Chinese cultural identity negatively affects the emotional attitude of health care in the traditional Chinese medicine.

#### 4.3.4. Mediation Effect of Demographic Characteristics

This study uses the software of Amos28.0 taking different demographic characteristics as control variables to test the modified structural equation model. The results show that gender, age, education, average monthly consumption level and occupation have no effect on the model. This shows that the modified structural equation model has certain universality.

## 5. Discussion and Enlightenment

Based on the “Dual Processing Theory” model, this study discusses the applicability of this theory in the context of consumption of health care in traditional Chinese medicine. The results show that performance expectation and the deep behavioral dimension of degree of Chinese cultural identity have a dual processing effect on the consumption attitude of health care in traditional Chinese medicine, which confirms the applicability of the theory.

### 5.1. Two Dimensions of Degree of Chinese Cultural Identity Significantly Affects the Consumption Attitude of Health Care for TCM, Respectively

The results of this study show that the two dimensions of degree of Chinese cultural identity significantly affect the consumption attitude of health care for TCM. The difference is that the surface cognitive dimension negatively affects the behavior attitude of health care for TCM, while the deep behavior dimension positively affects the consumption attitude of health care for TCM. Although Ding and Guan believe that Chinese culture is not only the basis for the formation of TCM theory, but also the driving force for the development of TCM theory [21]. In the process of formation and development, TCM has continuously absorbed the essence of Chinese traditional culture, such as Confucianism, Buddhism and Taoism, and formed the cultural characteristics of Chinese medicine. However, the results of this study show that the cognitive dimension of degree of Chinese cultural identity is not enough to have an impact on the consumption attitude of health care for TCM, and even have a negative impact. Only by deeply recognizing and acting on Chinese culture can it really have a positive impact on the consumption attitude of health care for TCM. This does not mean that there is something wrong with the Chinese culture on which health care fir TCM relies, nor does it mean that health care for TCM does not adapt to the market economy, but just means that health care for TCM are not worthy of the name. This dislocation between the superficial cognition of Chinese culture and the behavioral attitude towards health care for TCM leads to that only the actors who deeply identify with Chinese culture are the firm supporters of health care consumption for TCM.

### 5.2. Performance Expectation Has a Positive Impact on the Consumption Attitude of Health Care for TCM

The results of this study found that performance expectation (*β* =0.80) positively affects the consumption attitude of health care for TCM. Its influencing weight is higher than that of degree of Chinese cultural identity (*β* =0.06). It shows that consumers can treat health care for TCM rationally and attach great importance to the actual effect of health care for TCM. Previous studies in many fields have also shown that performance expectation can positively affect consumption attitudes. For example, the study of Ying finds that the most influential variables on consumers' willingness to use Alipay platform are performance expectation and social impact [22]. The data results of Chen and Jia also show that when the products or services observed or experienced by consumers meet performance expectation, consumers of risk averse will increase their willingness to consume products or services with high uncertainty, while consumers of risk preference will reduce their willingness to consume products or services with high uncertainty [23]. This shows that consumers of health care for TCM are likely to be risk averse, which is related to the fact that health care for TCM is a vital health product.

### 5.3. Degree of Chinese Cultural Identity and Performance Expectation Have a Positive Interaction on the Consumption Attitude of Health Care for TCM

The results of this study show that the higher the recognition of Chinese culture and the higher the performance expectation, the higher the consumer's attitude towards health care for TCM consumption. Based on the “Dual Processing Theory”, degree of Chinese cultural identity and performance expectation still have a positive impact on the game results of consumption attitude for health care of TCM. This is similar to the previous research results. Zhu and Wang found that variables such as performance expectation positively affect users' willingness to adopt the digital communication content of China's intangible cultural heritage [24]. Dong believes that when products and services are consumed, their value needs to be recognized. Culture is a necessary condition for participating in consumption activities. Through cultural identity, consumers' self-identity is brought, so as to realize the value-added effect of consumption identity with performance expectation [25]. In the process of health care for TCM consumption, performance expectation needs to be carried out in the context of Chinese cultural identity in order to realize the deep transformation from specific service to cultural identity. The unconscious, irrational and emotional power represented by Chinese culture makes the role of health care for TCM consumption clear. Consumers not only need the performance expectation of the service itself, but also need to interact with Chinese culture in consumption.

To sum up, this study believes that starting from the deep recognition of Chinese culture held by consumers in their hearts, we should constantly stimulate consumers' action cognition of Chinese culture, so as to positively affect the consumption attitude of health care for TCM. At the same time, we should standardize the whole industry of health care for TCM and improve the overall level of health care for TCM, so as to make consumers produce value interaction and emotional resonance in the consumption process of health care for TCM. It has a good enlightening effect on carrying forward TCM culture. Relationship culture is one of the traditional Chinese cultures, which is regarded as the core concept of understanding Chinese consumer behavior. In this cultural context, consumers' trading activities are often not simple economic interests, but also subtle and complex aspects such as human relations, reciprocal exchange, face problems and so on. Consumers' purchase behavior is often not just an economic transaction, but a kind of social interaction and relationship communication. Therefore, we can awaken the relationship marketing of consumers from the behavioral cognitive level, such as expanding the market scope by providing the business and social functions of health care for TCM.

## Figures and Tables

**Figure 1:** Model of Influencing Factors for Consumption Attitude of Health Care in Traditional Chinese Medicine.

**Figure 2:** Initial model.

**Figure 3:** Modified model.

**Table 1:** The operational definitions.

Variables	Coding	Measurement items
Degree of Chinese cultural identity	Q1	I think Chinese culture has a deep foundation.
	Q2	I think most of Chinese traditional culture is excellent.
	Q3	I like Chinese traditional clothes.
	Q4	I think Chinese traditional culture has a positive impact on my study, work and life.
	Q5	Traditional Chinese medicine is one of the representative elements of Chinese traditional culture.
	Q6	I am proud of Chinese traditional culture.
	Q7	I agree with the “unity of heaven and man” emphasized by Taoist culture.
	Q8	I think Chinese kung Fu is cool.
	Q9	I think traditional festivals are an important part of Chinese culture.
	Q10	I like traditional Chinese architecture.
	Q11	I often read ancient poetry, ancient prose and so on.
	Q12	I often visit museums related to Chinese traditional culture.
	Q13	When shopping, I will go to Chinese style shops.
	Q14	I often use my mobile phone to take photos for Chinese traditional style works of art, goods, etc.
	Q15	I will watch various activities related to Chinese traditional culture.
	Q16	I will collect Chinese traditional crafts.
	Q17	I will actively collect relevant knowledge of Chinese culture.
	Q18	I will take the initiative to spread Chinese culture.
Performance expectation	Q19	Health care in traditional Chinese medicine is very helpful to my daily work and life.
	Q20	Using the technology of health care in traditional Chinese medicine can effectively prevent diseases.
	Q21	Using the technology of health care in traditional Chinese medicine can maintain good health.
	Q22	Using the technology of health care in traditional Chinese medicine can improve the quality of life.
	Q23	Using the technology of health care in traditional Chinese medicine can reduce physical discomfort and the chance of illness.
Cognitive attitude	Q24	I understand the services of health care in traditional Chinese medicine.
	Q25	I have a new understanding of health care in traditional Chinese medicine.
Emotional attitude	Q26	I love health care in traditional Chinese medicine.
	Q27	I trust health care in traditional Chinese medicine.
Behavioral attitude	Q28	I have tried health care in traditional Chinese medicine.
	Q29	I will recommend to others to try health care in traditional Chinese medicine.

**Table 2:** Demographic characteristics of the samples (N =784).

Variable name	Classification	Frequency	Proportion	Variable name	Classification	Frequency	Proportion
Gender	Male	374	47.7%	Education	High school (technical secondary school) and below	26	3.3%
	Female	410	52.3%		Junior college	82	10.5%
Age	Under 18	222	28.3%		Undergraduate	384	49.0%
	18-30 years old	139	17.7%		Master	184	23.5%
	30-45 years old	127	16.2%		Doctor	108	13.8%
	45-60 years old	220	28.1%	Occupation	Student	112	14.3%
	Over 60 years old	76	9.7%		Private enterprise	193	24.6%
Level of average monthly consumption	Below 1500 yuan	156	19.9%		State-owned enterprise	195	24.9%
	1500-3000 below 1500 yuan	172	21.9%		Civil servant	133	17.0%
	3000-4500 below 1500 yuan	167	21.3%		Government-affiliated institutions	72	9.2%
	4500-6000 below 1500 yuan	68	8.7%		Self-employed	35	4.5%
	More than 6000 yuan	221	28.2%		Unemployed	8	1.0%
					Medical staff	34	4.4%
					Other	2	0.0%

**Table 3:** Confirmatory factor analysis.

Variables	Items	Parameter significance estimation					Convergent validity	Composite reliability
		Unstd	Std	S.E.	C.R.	*p*	AVE	C.R.
Surface cognition	Q1	1.000	0.802				0.661	0.951
	Q2	0.930	0.745	0.040	23.398	∗∗∗		
	Q3	0.971	0.779	0.039	24.813	∗∗∗		
	Q4	1.069	0.857	0.038	28.395	∗∗∗		
	Q5	0.955	0.765	0.039	24.250	∗∗∗		
	Q6	0.993	0.796	0.039	25.569	∗∗∗		
	Q7	1.112	0.891	0.037	30.061	∗∗∗		
	Q8	1.070	0.858	0.038	28.421	∗∗∗		
	Q9	0.961	0.771	0.039	24.467	∗∗∗		
	Q10	1.063	0.852	0.038	28.089	∗∗∗		

Deep behavior	Q11	1.000	0.705				0.589	0.918
	Q12	1.036	0.731	0.046	22.293	∗∗∗		
	Q13	1.179	0.832	0.053	22.383	∗∗∗		
	Q14	1.254	0.885	0.053	23.755	∗∗∗		
	Q15	1.235	0.871	0.053	23.411	∗∗∗		
	Q16	1.250	0.882	0.053	23.678	∗∗∗		
	Q17	0.888	0.626	0.053	16.876	∗∗∗		
	Q18	0.747	0.527	0.052	14.270	∗∗∗		

Performance expectation	Q19	1.000	0.880				0.874	0.972
	Q20	1.074	0.945	0.025	43.092	∗∗∗		
	Q21	1.094	0.963	0.024	45.348	∗∗∗		
	Q22	1.081	0.952	0.025	43.948	∗∗∗		
	Q23	1.058	0.932	0.026	41.483	∗∗∗		

Cognitive attitude	Q24	1.000	0.736				0.679	0.807
	Q25	1.227	0.903	0.046	26.443	∗∗∗		

Emotional attitude	Q26	1.000	0.896				0.789	0.882
	Q27	0.983	0.880	0.026	37.348	∗∗∗		

Behavioral attitude	Q28	1.000	0.814				0.740	0.850
	Q29	1.110	0.904	0.038	29.474	∗∗∗		

Note: ^∗^*p* < 0.05, ^∗∗^*p* < 0.01, and ^∗∗∗^*p* < 0.001.

**Table 4:** Model fitting index.

Index	Chi Square/DF	RMSEA	GFI	AGFI	NFI	CFI	TLI	IFI
Value	4.897	0.071	0.855	0.824	0.928	0.942	0.934	0.942

**Table 5:** Path analysis.

Path	Estimate	S.E.	C.R.	P
Surface cognition⇄performance expectation	0.582	0.039	14.921	∗∗∗
Deep behavior⇄performance expectation	0.469	0.035	13.415	∗∗∗
Surface cognition⇄deep behavior	0.523	0.036	14.392	∗∗∗
Surface cognition→cognitive attitude	-0.035	0.040	-0.875	0.382
Surface cognition→emotional attitude	-0.036	0.048	-0.784	0.455
Surface cognition→deep behavior	-0.153	0.054	-2.812	0.005
Deep behavior→cognitive attitude	0.096	0.043	2.247	0.025
Deep behavior→emotional attitude	0.105	0.052	2.029	0.042
Deep behavior→behavioral attitude	0.218	0.058	3.751	∗∗∗
Performance expectation→cognitive attitude	0.628	0.035	18.052	∗∗∗
Performance expectation→emotional attitude	0.819	0.032	25.243	∗∗∗
Performance expectation→behavioral attitude	0.679	0.037	18.200	∗∗∗

Note: ∗*p* < 0.05, ∗∗*p* < 0.01, ∗∗∗*p* < 0.001.

## Data Availability

The data used to support the findings of this study are available from the corresponding author upon request.
